# A novel live cell assay to measure diacylglycerol lipase α activity

**DOI:** 10.1042/BSR20160073

**Published:** 2016-05-06

**Authors:** Praveen K. Singh, Rachel Markwick, Fiona V. Howell, Gareth Williams, Patrick Doherty

**Affiliations:** * Wolfson Centre for Age-Related Diseases, King's College London, SE1 9RT, U.K.

**Keywords:** diacylglycerol lipase α (DAGLα), 6,8-difluoro-4-methylumbelliferyl octanoate (DiFMUO), live cell assay, *p*-nitrophenyl butyrate (PNPB)

## Abstract

Diacylglycerol lipase α (DAGLα) hydrolyses DAG to generate the principal endocannabinoid (eCB) 2-arachidonoylglycerol (2-AG) in the central nervous system. DAGLα dependent cannabinoid (CB) signalling has been implicated in numerous processes including axonal growth and guidance, adult neurogenesis and retrograde signalling at the synapse. Recent studies have implicated DAGLα as an emerging drug target for several conditions including pain and obesity. Activity assays are critical to the drug discovery process; however, measurement of diacylglycerol lipase (DAGL) activity using its native substrate generally involves low-throughput MS techniques. Some relatively high-throughput membrane based assays utilizing surrogate substrates have been reported, but these do not take into account the rate-limiting effects often associated with the ability of a drug to cross the cell membrane. In the present study, we report the development of a live cell assay to measure DAGLα activity. Two previously reported DAGLα surrogate substrates, *p*-nitrophenyl butyrate (PNPB) and 6,8-difluoro-4-methylumbelliferyl octanoate (DiFMUO), were evaluated for their ability to detect DAGLα activity in live cell assays using a human cell line stably expressing the human DAGLα transgene. Following optimization, the small molecule chromogenic substrate PNPB proved to be superior by providing lower background activity along with a larger signal window between transfected and parental cells when compared with the fluorogenic substrate DiFMUO. The assay was further validated using established DAGL inhibitors. In summary, the live cell DAGLα assay reported here offers an economical and convenient format to screen for novel inhibitors as part of drug discovery programmes and compliments previously reported high-throughput membrane based DAGL assays.

## INTRODUCTION

The diacylglycerol lipases (DAGLs), diacylglycerol lipase α (DAGLα) and diacylglycerol lipase β (DAGLβ), hydrolyse DAG to generate 2-arachidonoylglycerol (2-AG) for endocannabinoid (eCB) signalling which has been implicated in numerous important processes including axonal growth and guidance during development [1–6], synaptic plasticity in the form of retrograde synaptic transmission [7,8] and adult neurogenesis in the hippocampus and subventricular zone [1,7,9,10]. 2-AG generated by the DAGLs also acts as a substrate for monoacylglycerol lipase to maintain arachidonic acid (AA) levels in various tissues [7,11,12].

The DAGLs are emerging therapeutic targets for a range of conditions including fragile X syndrome, pain, inflammatory diseases and obesity [13–16]. Furthermore, drugs modulating other steps of eCB signalling have shown beneficial effects in obesity [17–20], pain [21,22], Alzheimer's disease [23] and Parkinson's disease [24]. DAGLα in particular is responsible for almost all of the 2-AG in the central nervous system and for retrograde signalling at the synapses via the cannabinoid (CB) receptors [7,8]. Selectively targeting DAGLα may therefore prove fruitful for the treatment of certain conditions as it has the potential to avoid the adverse psychiatric effects observed when targeting the cannabinoid receptor 1 (CB1) receptor [25].

As evidenced by previous and recent publications, there are several ongoing drug discovery efforts related to the DAGLs [13,16,26–35]. These studies have largely utilized assays employing isolated membranes (or lysates) overexpressing the DAGLs. At present, there are no simple assays that measure the activity of the human DAGLs in a live cell context. Such assays play an important role in drug discovery efforts and are particularly useful as they take into account the cell permeability of inhibitors and also present the target in a relatively native as opposed to isolated environment [36,37]. In the present study, we have generated a human U2OS cell line stably expressing an epitope tagged human DAGLα transgene. Two commercially available DAGLα surrogate substrates [26], namely *p*-nitrophenyl butyrate (PNPB) and 6,8-difluoro-4-methylumbelliferyl octanoate (DiFMUO) were evaluated in live cell assays using the cell line to determine if we could measure activity of the DAGLα transgene in intact cells. The small chromogenic molecule PNPB was found to be a suitable substrate, showing a larger difference in activity between transfected and parental cells along with lower background activity when compared with the fluorogenic substrate DiFMUO. The specificity of the response was confirmed using several established DAGL inhibitors. The live cell assay for DAGLα described here offers an economical and convenient format to screen for novel cell-permeant inhibitors as a complement to currently available membrane based assays.

## MATERIALS AND METHODS

### Reagents

All reagents were purchased from Sigma–Aldrich unless otherwise stated.

### Generation of the V5α11 cell line

In order to express DAGLα with a V5 tag (C-terminal), full-length human DAGLα [2] was cloned into the pCDNA6.2/V5-DEST vector (Invitrogen). The construct was transfected (Lipofectamine 2000, Invitrogen) into a human U2OS osteosarcoma cell line (Tango™ CNR1-bla U2OS cells from Invitrogen) that for the purpose of future studies also expresses a CB1 reporter construct. Selection of stable transfected clones was performed using blasticidin (4 μg/ml). Several clones were repeatedly screened by Western blotting and immunocytochemical analyses using a V5 antibody (mouse, Invitrogen) following which the cell line stably expressing DAGLα with a C-terminal V5 tag (DAGLα-V5) (V5α11) was established.

### Membrane preparation

Membranes were prepared following the method described by Pedicord et al. [26]. Briefly, V5α11 or tango (parental) cells (∼90% confluent) cultured in 10 cm dishes were washed with PBS following which the cells were scraped in 1 ml (per dish) of lysis buffer (20 mM HEPES, pH 7.0, 2 mM DTT, 0.25 M sucrose, 10 mM NaF, 1 mM Na_3_VO_4_ and 1× Roche ‘Complete™’ protease inhibitor). The cell suspensions were collected and homogenized on ice using a Polytron (PT 1200 E) homogenizer (three 7 s bursts at the maximum setting with 30 s interval in between). The homogenates were centrifuged at 100000 ***g*** for 30 min at 4°C following which the supernatants were discarded. The pellets (membrane preparations) were resuspended in 200 μl of sucrose free lysis buffer using the Polytron homogenizer and stored at–80°C.

### Immunocytochemistry

Cells were first seeded on to polylysine coated coverslips at a density of 10000/well and cultured overnight following which they were fixed in 4% paraformaldehyde for 30 min. The fixed cells were washed with PBS and then permeabilized for 10 min using 0.2% Triton X-100-PBS. The permeabilized cells were washed with PBS and then blocked for 30 min using the block solution (1% BSA–PBS). The cells were then incubated with the V5 primary antibody (mouse, Invitrogen, diluted 1/1000 in block solution) for 1 h at room temperature, washed with PBS and then incubated for 1 h with the AlexaFluor 488 secondary antibody (mouse, Invitrogen, diluted 1/2000 in block solution) and the nuclear stain Hoechst 33258 (Invitrogen, diluted 1/10000 in block solution). Finally, the cells were washed with PBS and the coverslips were mounted on to microscope slides. The Carl Zeiss LSM 710 microscope and the Carl Zeiss Zen software (version 1.0.1.0) were used to capture images of the immunostained cells.

### Western blotting

V5α11 or tango membranes were diluted using 5× SDS protein loading buffer and water to a concentration of 1 μg/μl. Diluted samples were denatured by boiling for 5 min. Ten micrograms of the denatured samples were loaded on to Tris-glycine gels (4% stacking and 10% resolving) and resolved at a setting of 100 V for ∼2 h. Western blotting was performed using nitrocellulose membranes (GE healthcare) and a wet transfer method (1 h at 100 V and 4°C). Membranes were blocked in PBS 5% milk (1 h at room temperature) and then incubated with the primary V5 antibody [diluted in PBS 0.1% Tween (PBST) 2% milk] overnight at 4°C. The membranes were then washed in PBST and incubated with the mouse IR-Dye 680 secondary antibody (LI-COR, diluted 1/5000 in PBST 2% milk) for 1 h at room temperature. Finally, the membranes were washed in PBST (4×) and then PBS (1×). The Odyssey imaging system (LI-COR) was used to visualize the membranes. β-Actin was also detected as a loading control.

### Membrane assays

All membrane assays were carried out in 96-well clear polypropylene plates following a previously published method with some modifications [26]. Membranes were first diluted in assay buffer (4× FAC, i.e. final assay concentration) following which 50 μl/well was dispensed. Fifty microlitres of assay buffer or 50 μl of inhibitor (diluted to 4× FAC using assay buffer) was then added to the membranes. Membranes were typically incubated with the inhibitors in the plates for 5 min at room temperature. Substrate was first diluted in DMSO to 40× FAC and then to 2× FAC using the assay buffer without DMSO. Hundred microlitres/well of the substrate solution was dispensed and the plates were read immediately. For the PNPB assay, 50 mM HEPES pH 7.5 and 5% DMSO was used as the assay buffer and reactions were monitored by measuring the optical density at 400 nm (OD400) every 12 s for 30 min using a Spectramax plate reader (Molecular Devices). For the DiFMUO assay, 50 mM MES pH 6.5 and 5% DMSO was used as the assay buffer and the reactions were monitored by measuring the fluorescence (excitation 360 nm, emission 450 nm) every 30 s for 30 min using the FlexStation (Molecular Devices). Typically, FACs were 12.5 μg/ml membranes, 250 μM PNPB or 10 μM DiFMUO, and 5% DMSO in a total assay volume of 200 μl. Activity was determined by calculating the reaction rates over the first 10 min (linear) using three replicate wells.

### Live cell assay

Cells were seeded at a density of 40000/well (96-well plates) in FreeStyle media (Invitrogen) and maintained overnight. Prior to assaying, the media were discarded and the cells were washed with the assay buffer (50 mM HEPES, pH 7.5 for the PNPB assay and 50 mM MES, pH 6.5 for the DiFMUO assay). One hundred microlitres of inhibitor (2× FAC) or assay buffer was then added to the wells following which the plate was incubated for 5 min. One hundred microlitres of substrate (diluted to 100× FAC in DMSO and then to 2× FAC in assay buffer) was then added to each well and the activity was measured as described for the corresponding membrane assay (six replicate wells). Typically, the total assay volume was 200 μl containing 1% DMSO and either 500 μM PNPB or 10 μM DiFMUO.

## RESULTS

The U2OS cell line stably expressing DAGLα-V5 (V5α11) was established to support the development of a DAGLα live cell assay. Stable expression of DAGLα-V5 was confirmed beyond 30 passages in this cell line by both Western and immunocytochemistry analyses using a V5 antibody (Figure 1). In order to test the activity of DAGLα-V5 expressed in the V5α11cell line, activity of membranes derived from parental and V5α11 cells was measured using two previously reported DAGLα surrogate substrates (DiFMUO and PNPB) [26]. A relatively modest but significant 1.6-fold difference in activity was detected between the V5α11 and parental membranes using the larger fluorogenic DiFMUO as the substrate (Figure 2A). This ‘window’ was achieved following optimization of various parameters including assay buffer constituents and the substrate and membrane concentrations. Notably, this difference in activity was inhibited by the DAGL inhibitor tetrahydrolipstatin (THL) which provided a slightly improved 1.8-fold difference in THL sensitive activity of the two membranes.

**Figure 1:** Stable expression of human DAGLα-V5 in the V5α11 cell line DAGLα-V5 expression in the V5α11 cell line was periodically monitored by Western and immunocytochemical analyses using a V5 antibody. A representative image demonstrating the stable and clonal expression of DAGLα-V5 in fixed V5α11 cells immunostained with a V5 antibody (green) and the nuclear stain Hoechst (blue) is presented above along with parental cells as a negative control (**A**). Western analyses using V5α11 membranes (and parental membranes as a negative control) and a V5 antibody revealed DAGLα-V5 expression at a size close to the predicted molecular mass (120 kDa) (**B**).

**Figure 2:** Characterizing DAGLα activity in the V5α11 membranes using DiFMUO and PNPB Activities of V5α11 and parental membranes were measured using surrogate substrates. Membranes (12.5 μg/ml) were first incubated in the presence or absence of THL (1 μM) for 5 min following which the activity was measured using 10 μM DiFMUO (mean±S.E.M., *n*=7) (**A**) or 250 μM PNPB (mean±S.E.M.; V5α11, *n*=10; parental, *n*=13) (**B**). The difference in PNPB hydrolytic activity between the membranes was inhibited by three different DAGL inhibitors (OMDM-188, THL and RHC-80267) (mean of three wells±S.E.M.) (**C**). The reaction rates were calculated over the first 10 min; **P<0.01, ***P< 0.001 (two-tailed *t* test).

On the other hand, the V5α11 cell line showed 6-fold greater PNPB hydrolysis activity than parental membranes; this difference was enhanced to 11-fold when considering the THL sensitive activity (Figure 2B). These results indicate that PNPB is a superior substrate for the measurement of DAGLα activity when using the V5α11 membranes. The relatively low PNPB hydrolysis activity in the parental membranes (compared with V5α11) validated the V5α11 membranes as a tool to screen for DAGLα inhibitors. IC_50_s of three DAGL inhibitors, OMDM-188 (2.1±0.15 nM), THL (5.3±0.23 nM) and RHC-80267 (28.8±11.1 μM) were determined in the assay (Figure 2C). The results are in agreement with previous studies; OMDM-188 has been reported to be the more potent of the three DAGL inhibitors whereas RHC-80267 has been reported to be the least potent [26,38,39].

Cell based assays in conjunction with biochemical assays are a critical part of drug discovery programmes. Having identified significant differences between the activity of the V5α11 membranes using PNPB and DiFMUO, we next investigated whether these surrogate substrates could also be used as part of DAGLα live cell assays. In order to assess whether background activity due to cytoplasmic enzymes could prove to be problematic, we first tested the activity of crude cell homogenates prepared from V5α11 and parental cells using the substrates. Unsurprisingly, only a 1.5-fold difference was observed when comparing activity of the homogenates using DiFMUO as the substrate (Supplementary Figure S1A) and despite optimization of various parameters, only a modest (but significant) 1.3-fold (1.4-fold THL sensitive) difference was observed when measuring the activity in intact cells (Figure 3A).

**Figure 3:** Live cell based assays to measure DAGLα activity V5α11 or parental cells (40000 cells/well, seeded and maintained overnight in 96-well plates) were washed and then incubated in the presence or absence of THL (25 μM) for 5 min. The activity was then measured using 10 μM DiFMUO (mean±S.E.M.; V5α11, *n*=16; parental, *n*=22) (**A**) or 500 μM PNPB (mean±S.E.M., *n*=9) (**B**). The difference in PNPB hydrolytic activity between the two cell lines was inhibited by the DAGL inhibitors RHC-80267 and THL (six replicate wells±S.E.M.) (**C**). The reaction rates were calculated over the first 10 min; ***P<0.001 (two-tailed *t* test).

On the other hand, encouragingly, 4-fold greater activity was observed in V5α11 crude homogenates when compared with parental homogenates using PNPB indicating that potential background hydrolysis by cytoplasmic enzymes was relatively low compared with DAGLα-V5 activity when using this substrate (Supplementary Figure S1B). Following optimization of assay buffer constituents (Supplementary Figures S1C and S1D), substrate concentration (Supplementary Figure S1E) and cell numbers (Supplementary Figure S1F), 2.1-fold greater PNPB hydrolysis activity was observed in the V5α11 cells compared with the parental cells when the substrate was added to intact cells. This difference in activity was inhibited by THL (Figure 3B). IC_50_s of THL and RHC-80267 (IC_50_s 31.8±4.1 nM and 5.8±0.2 μM respectively) were also determined using this assay (Figure 3C). When subtracting the background activity seen in the presence of THL, the difference in activity between the two cell lines using PNPB was much higher at 3.5-fold. Thus, we conclude that PNPB is a more suitable substrate to measure DAGLα activity in both membrane and live cell assays.

## DISCUSSION

The DAGLs have been implicated in a range of diseases and therefore have previously and recently been the focus of several studies aiming to discover novel inhibitors of these enzymes [13–16,27,30,31]. In support of such studies, numerous assays that can measure DAGL activity in isolated membranes and/or lysates have been reported. These include low-throughput MS based native substrate assays that employ synthetic DAG as a substrate coupled with the measurement of 2-AG as the product [40,41]. Low-throughput assays that utilize radiolabelled substrates or activity based probes have also been described [2,13,29–31,41]. Previously, relatively higher throughput surrogate substrate (fluorogenic or chromogenic), FRET (using ether lipid reporters) and native substrate (coupled enzyme) assays of particular utility for drug discovery programmes have been reported [26,28,29]. However, at present there are no simple assays that measure the activity of the DAGLs in a live cell context. Live cell assays are clearly of considerable value as they will act as a filter for drugs that have limited access to the cytoplasm in cells, and efficacy measurements will take into account this important variable. Furthermore, they present the target in a relatively native environment.

As a complement to the above mentioned assays, we report here the development of a simple live cell assay to measure DAGLα activity. This live cell assay does not involve a cell lysis step and employs the relatively economical chromogenic DAGL surrogate substrate PNPB [26]. Firstly, by establishing a U2OS cell line that stably and robustly expresses the DAGLα transgene, we have developed a tool to directly study DAGLα catalytic activity (using membranes or cells). Notably, the parental human cell line has also been previously modified to express a CB1 reporter construct (Tango™ CNR1-bla U2OS cells from Invitrogen) and therefore the V5α11 cells also have the potential to measure DAGL-dependent CB1 activation. In the present study, the difference in activity between the V5α11 and parental cells (or membranes) was higher when using the smaller chromogenic PNPB substrate (2.1- to 3.5-fold in the cellular assay, 6- to 11-fold in the membrane assay) in comparison with the larger fluorogenic substrate DiFMUO (≤1.8-fold). Higher background enzymatic activity in the parental cells and/or generally lower DAGLα activity against DiFMUO when compared with PNPB may account for these differences. Pedicord et al. [26] suggested that DiFMUO may access DAGLα through the membrane whereas PNPB may access this enzyme through the aqueous phase in which case DiFMUO membrane diffusion rates could prove to be rate limiting and explain the differences observed in activity. DiFMUO (338 Da) is also a larger molecule when compared with PNPB (209 Da) and this may also influence DAGLα activity against this substrates as the active site of lipases are regulated by a displaceable lid like structure [42,43].

The DAGLα-V5 PNPB live cell assay described here provided a THL sensitive signal window of ∼3.4-fold but the difference in activity when comparing the two cell lines was considerably lower (2-fold) when including the THL insensitive activity. It is unlikely that endogenous DAGLα (or DAGLβ) are major contributors towards the PNPB hydrolytic activity observed in the parental cells for the following reason. As the DAGLs are membrane proteins and both are inhibited by THL, any endogenous DAGL activity would have contributed towards the THL sensitive activity measured in the parental membranes which was however much lower than the activity attributed to the overexpressed DAGLα-V5 (10-fold greater). This is further corroborated by the fact that DAGLα-V5 expression is 10- to 15-fold greater than endogenous DAGLα or DAGLβ [reverse transcription polymerase chain reaction (RT-PCR) analysis; results not shown] and this along with the assay data indicate that cytoplasmic lipases/hydrolases are likely contributors towards the higher PNPB hydrolytic activity observed in the parental cells when compared with membranes. Candidate ‘interfering’ lipases include the hormone sensitive lipase and lipoprotein lipase which have reported PNPB hydrolytic activity [44,45]. In this context, as PNPB is a surrogate DAGL substrate and is also hydrolysed by some other lipases/hydrolases, it is unlikely that PNPB can be used to measure endogenous DAGLα activity in primary cells although it will still be tempting to measure PNPB hydrolytic activity in primary cells that are ‘high’ expressers of DAGLα (e.g. neurons) in conjunction with recently developed specific DAGL inhibitors in order to determine the contribution of DAGLα towards the measured activity [2,13,27,30]. In general though, PNPB is more suitable for measuring DAGLα activity in assays employing overexpressing cell lines as described here where the activity of the recombinant enzyme is several fold higher than the endogenous and/or background activities. Although the use of whole cells (or membranes as opposed to purified protein) preclude *K*_cat_ calculations, as is the case with other published DAGL assays [2,13,26,28,29], the assay reported here is continuous and employs a chromogenic substrate and so can be used to monitor inhibition kinetics (time course; different inhibitor and substrate concentrations) in a cellular environment [26]. Improving the signal window of the assay would be beneficial for such studies and would entail three approaches–(1) Increasing DAGLα-V5 activity which could be achieved by generating cell lines expressing higher amounts of DAGLα-V5. (2) Reducing non-DAGLα enzymatic activity which could be achieved by employing pharmacological tools to identify candidate ‘interfering’ enzymes and then genetic tools to disrupt their expression/activity. (3) Reducing non-enzymatic activity by further optimization of assay conditions/reagents, e.g. culture conditions, choice of plates, buffer components [46].

The DAGLα-V5 PNPB live cell assay described here could be applied as a primary or secondary assay for DAGLα drug discovery programmes or as a selectivity assay for DAGLβ drug discovery programmes. In this context, DAGLα is responsible for almost all of the 2-AG in the brain and for CB1 receptor mediated retrograde signalling at the synapses [7,8]. Selectively targeting DAGLα may therefore prove fruitful for the treatment of certain conditions (e.g. obesity) as it has the potential to avoid the adverse psychiatric effects observed when targeting the CB1 receptor [16,25]. On the other hand, there is growing interest in DAGLβ as a target for inflammatory diseases and maintaining selectivity of DAGLβ inhibitors over DAGLα may help avoid unwanted modulation of synaptic signalling [13]. Similarly, the assay described here could also be applied as a selectivity assay for modulators targeting other members of the eCB system or closely related lipases.

In conclusion, the DAGLα overexpressing V5α11 cells and the chromogenic surrogate substrate, PNPB, provide the basis for relatively simple assays that can characterize the ability of drugs to inhibit the activity of this enzyme in membranes and in a live cell context with utility as primary, secondary and selectivity assays for drug discovery programmes.

## Abbreviations

AA: arachidonic acid
2-AG: 2-arachidonoylglycerol
CB: cannabinoid
CB1: cannabinoid receptor 1
DAG: diacylglycerol
DAGL: diacylglycerol lipase
DAGLα: diacylglycerol lipase α
DAGLα: DAGLα with a C-terminal V5 tag
DAGLβ: diacylglycerol lipase β
DiFMUO: 6,8-difluoro-4-methylumbelliferyl octanoate
eCB: endocannabinoid
FAC: final assay concentration
OD400: optical density at 400 nm
PBST: phosphate buffered saline 0.1% Tween
PNPB: *p*-nitrophenyl butyrate
RT-PCR: reverse transcription polymerase chain reaction
THL: tetrahydrolipstatin

## References

[1] Oudin M.J., Hobbs C., Doherty P. (2011). DAGL-dependent endocannabinoid signalling: roles in axonal pathfinding, synaptic plasticity and adult neurogenesis. Eur. J. Neurosci..

[2] Bisogno T., Howell F., Williams G., Minassi A., Cascio M.G., Ligresti A., Matias I., Schiano-Moriello A., Paul P., Williams E.J. (2003). Cloning of the first sn1-DAG lipases points to the spatial and temporal regulation of endocannabinoid signaling in the brain. J. Cell Biol..

[3] Williams E.J., Walsh F.S., Doherty P. (2003). The FGF receptor uses the endocannabinoid signaling system to couple to an axonal growth response. J. Cell Biol..

[4] Wu C.S., Zhu J., Wager-Miller J., Wang S., O'Leary D., Monory K., Lutz B., Mackie K., Lu H.C. (2010). Requirement of cannabinoid CB(1) receptors in cortical pyramidal neurons for appropriate development of corticothalamic and thalamocortical projections. Eur. J. Neurosci..

[5] Mulder J., Aguado T., Keimpema E., Barabas K., Ballester Rosado C.J., Nguyen L., Monory K., Marsicano G., Di Marzo V., Hurd Y.L. (2008). Endocannabinoid signaling controls pyramidal cell specification and long-range axon patterning. Proc. Natl. Acad. Sci. U.S.A..

[6] Watson S., Chambers D., Hobbs C., Doherty P., Graham A. (2008). The endocannabinoid receptor, CB1, is required for normal axonal growth and fasciculation. Mol. Cell Neurosci..

[7] Gao Y., Vasilyev D.V., Goncalves M.B., Howell F.V., Hobbs C., Reisenberg M., Shen R., Zhang M.Y., Strassle B.W., Lu P. (2010). Loss of retrograde endocannabinoid signaling and reduced adult neurogenesis in diacylglycerol lipase knock-out mice. J. Neurosci..

[8] Tanimura A., Yamazaki M., Hashimotodani Y., Uchigashima M., Kawata S., Abe M., Kita Y., Hashimoto K., Shimizu T., Watanabe M. (2010). The endocannabinoid 2-arachidonoylglycerol produced by diacylglycerol lipase alpha mediates retrograde suppression of synaptic transmission. Neuron.

[9] Oudin M.J., Gajendra S., Williams G., Hobbs C., Lalli G., Doherty P. (2011). Endocannabinoids regulate the migration of subventricular zone-derived neuroblasts in the postnatal brain. J. Neurosci..

[10] Goncalves M.B., Suetterlin P., Yip P., Molina-Holgado F., Walker D.J., Oudin M.J., Zentar M.P., Pollard S., Yáñez-Muñoz R.J., Williams G. (2008). A diacylglycerol lipase-CB2 cannabinoid pathway regulates adult subventricular zone neurogenesis in an age-dependent manner. Mol. Cell Neurosci..

[11] Nomura D.K., Hudak C.S., Ward A.M., Burston J.J., Issa R.S., Fisher K.J., Abood M.E., Wiley J.L., Lichtman A.H., Casida J.E. (2008). Monoacylglycerol lipase regulates 2-arachidonoylglycerol action and arachidonic acid levels. Bioorg. Med. Chem. Lett..

[12] Nomura D.K., Blankman J.L., Simon G.M., Fujioka K., Issa R.S., Ward A.M., Cravatt B.F., Casida J.E. (2008). Activation of the endocannabinoid system by organophosphorus nerve agents. Nat. Chem. Biol..

[13] Hsu K.L., Tsuboi K., Adibekian A., Pugh H., Masuda K., Cravatt B.F. (2012). DAGLbeta inhibition perturbs a lipid network involved in macrophage inflammatory responses. Nat. Chem. Biol..

[14] Jung K.M., Sepers M., Henstridge C.M., Lassalle O., Neuhofer D., Martin H., Ginger M., Frick A., DiPatrizio N.V., Mackie K. (2012). Uncoupling of the endocannabinoid signalling complex in a mouse model of fragile X syndrome. Nat. Commun..

[15] Gregg L.C., Jung K.M., Spradley J.M., Nyilas R., Suplita R.L., Zimmer A., Watanabe M., Mackie K., Katona I., Piomelli D., Hohmann A.G. (2012). Activation of type 5 metabotropic glutamate receptors and diacylglycerol lipase-alpha initiates 2-arachidonoylglycerol formation and endocannabinoid-mediated analgesia. J. Neurosci..

[16] Bisogno T., Mahadevan A., Coccurello R., Chang J.W., Allarà M., Chen Y., Giacovazzo G., Lichtman A., Cravatt B., Moles A., Di Marzo V. (2013). A novel fluorophosphonate inhibitor of the biosynthesis of the endocannabinoid 2-arachidonoylglycerol with potential anti-obesity effects. Br. J. Pharmacol..

[17] Kunos G., Tam J. (2011). The case for peripheral CB(1) receptor blockade in the treatment of visceral obesity and its cardiometabolic complications. Br. J. Pharmacol..

[18] Marco E.M., Romero-Zerbo S.Y., Viveros M.P., Bermudez-Silva F.J. (2012). The role of the endocannabinoid system in eating disorders: pharmacological implications. Behav. Pharmacol..

[19] McLaughlin P.J. (2012). Reports of the death of CB1 antagonists have been greatly exaggerated: recent preclinical findings predict improved safety in the treatment of obesity. Behav. Pharmacol..

[20] Silvestri C., Di Marzo V. (2012). Second generation CB1 receptor blockers and other inhibitors of peripheral endocannabinoid overactivity and the rationale of their use against metabolic disorders. Expert. Opin. Investig. Drugs.

[21] Zogopoulos P., Vasileiou I., Patsouris E., Theocharis S.E. (2013). The role of endocannabinoids in pain modulation. Fundam. Clin. Pharmacol..

[22] Guindon J., Hohmann A.G. (2009). The endocannabinoid system and pain. CNS Neurol. Disord. Drug Targets..

[23] Piro J.R., Benjamin D.I., Duerr J.M., Pi Y., Gonzales C., Wood K.M., Schwartz J.W., Nomura D.K., Samad T.A. (2012). A dysregulated endocannabinoid-eicosanoid network supports pathogenesis in a mouse model of Alzheimer's disease. Cell Rep..

[24] Nomura D.K., Morrison B.E., Blankman J.L., Long J.Z., Kinsey S.G., Marcondes M.C., Ward A.M., Hahn Y.K., Lichtman A.H., Conti B., Cravatt B.F. (2011). Endocannabinoid hydrolysis generates brain prostaglandins that promote neuroinflammation. Science.

[25] Moreira F.A., Crippa J.A.S. (2009). The psychiatric side-effects of rimonabant. Rev. Bras. Psiquiatr..

[26] Pedicord D.L., Flynn M.J., Fanslau C., Miranda M., Hunihan L., Robertson B.J., Pearce B.C., Yu X.C., Westphal R.S., Blat Y. (2011). Molecular characterization and identification of surrogate substrates for diacylglycerol lipase alpha. Biochem. Biophys. Res. Commun..

[27] Appiah K.K., Blat Y., Robertson B.J., Pearce B.C., Pedicord D.L., Gentles R.G., Yu X.C., Mseeh F., Nguyen N., Swaffield J.C. (2014). Identification of small molecules that selectively inhibit diacylglycerol lipase-α activity. J. Biomol. Screen..

[28] van der Wel T, Janssen F.J., Baggelaar M.P., Deng H., den Dulk H., Overkleeft H.S., van der Stelt M. (2015). A natural substrate-based fluorescence assay for inhibitor screening on diacylglycerol lipase α. J. Lipid. Res..

[29] Johnston M., Bhatt S.R., Sikka S., Mercier R.W., West J.M., Makriyannis A., Gatley S.J., Duclos R.I. (2012). Assay and inhibition of diacylglycerol lipase activity. Bioorg. Med. Chem. Lett..

[30] Baggelaar M.P., Janssen F.J., van Esbroeck A.C.M., den Dulk H., Allarà M., Hoogendoorn S., McGuire R., Florea B.I., Meeuwenoord N., van den Elst H. (2013). Development of an activity-based probe and *in silico* design reveal highly selective inhibitors for diacylglycerol lipase-α in brain. Angew. Chem. Int. Ed. Engl..

[31] Hsu K.L., Tsuboi K., Whitby L.R., Speers A.E., Pugh H., Inloes J., Cravatt B.F. (2013). Development and optimization of piperidyl-1,2,3-triazole ureas as selective chemical probes of endocannabinoid biosynthesis. J. Med. Chem..

[32] Janssen F.J., Deng H., Baggelaar M.P., Allarà M., van der Wel T., den Dulk H., Ligresti A., van Esbroeck A.C., McGuire R., Di Marzo V. (2014). Discovery of glycine sulfonamides as dual inhibitors of sn-1-diacylglycerol lipase α and α/β-hydrolase domain 6. J. Med. Chem..

[33] Janssen F.J., Baggelaar M.P., Hummel J.J.A., Overkleeft H.S., Cravatt B.F., Boger D.L., van der Stelt M. (2015). Comprehensive analysis of structure activity relationships of α-ketoheterocycles as sn-1-diacylglycerol lipase α inhibitors. J. Med. Chem..

[34] Baggelaar M.P., Chameau P.J.P., Kantae V., Hummel J., Hsu K.L., Janssen F., van der Wel T., Soethoudt M., Deng H., den Dulk H. (2015). Highly selective, reversible inhibitor identified by comparative chemoproteomics modulates diacylglycerol lipase activity in neurons. J. Am. Chem. Soc..

[35] Ogasawara D., Deng H., Viader A., Baggelaar M.P., Breman A., den Dulk H., van den Nieuwendijk A.M., Soethoudt M., van der Wel T., Zhou J. (2015). Rapid and profound rewiring of brain lipid signaling networks by acute diacylglycerol lipase inhibition. Proc. Natl. Acad. Sci. U.S.A..

[36] Moore K., Rees S. (2001). Cell-based versus isolated target screening: how lucky do you feel?. J. Biomol. Screen..

[37] Fox S., Farr-Jones S., Sopchak L., Boggs A., Nicely H.W., Khoury R., Biros M. (2006). High-throughput screening: update on practices and success. J. Biomol. Screen..

[38] Bisogno T., Cascio M.G., Saha B., Mahadevan A., Urbani P., Minassi A., Appendino G., Saturnino C., Martin B., Razdan R., Di Marzo V. (2006). Development of the first potent and specific inhibitors of endocannabinoid biosynthesis. Biochim. Biophys. Acta.

[39] Ortar G., Bisogno T., Ligresti A., Morera E., Nalli M., Di Marzo V. (2008). Tetrahydrolipstatin analogues as modulators of endocannabinoid 2-arachidonoylglycerol metabolism. J. Med. Chem..

[40] Jung K.M., Astarita G., Zhu C., Wallace M., Mackie K., Piomelli D. (2007). A key role for diacylglycerol lipase-alpha in metabotropic glutamate receptor-dependent endocannabinoid mobilization. Mol. Pharmacol..

[41] Hoover H.S., Blankman J.L., Niessen S., Cravatt B.F. (2008). Selectivity of inhibitors of endocannabinoid biosynthesis evaluated by activity-based protein profiling. Bioorg. Med. Chem. Lett..

[42] Nardini M., Dijkstra B.W. (1999). Alpha/beta hydrolase fold enzymes: the family keeps growing. Curr. Opin. Struct. Biol..

[43] Holmquist M. (2000). Alpha/Beta-hydrolase fold enzymes: structures, functions and mechanisms. Curr. Protein Pept. Sci..

[44] Shirai K., Jackson R.L., Quinn D.M. (1982). Reciprocal effect of apolipoprotein C-II on the lipoprotein lipase-catalyzed hydrolysis of p-nitrophenyl butyrate and trioleoylglycerol. J. Biol. Chem..

[45] Laurell H., Contreras J.A., Castan I., Langin D., Holm C. (2000). Analysis of the psychrotolerant property of hormone-sensitive lipase through site-directed mutagenesis. Protein Eng..

[46] Zhang Z., Guan N., Li T., Mais D.E., Wang M. (2012). Quality control of cell-based high-throughput drug screening. Acta Pharm. Sinica B.

